This article has been retracted.

# A Study on the Impact of Digital Finance on Regional Productivity Growth Based on Artificial Neural Networks

**DOI:** 10.1155/2022/7665954

**Published:** 2022-05-31

**Authors:** Jia Li, Fangcheng Sun, Meng Li

**Affiliations:** ^1^Research Center for Economy of Upper Reaches of the Yangtze River, Chongqing Technology and Business University, Chongqing 400060, China; ^2^School of Tourism and Event Management of Chongqing University of Arts and Sciences, Chongqing 402160, China

## Abstract

The relationship between financial development and economic growth has become a hot topic in recent years and for China, which is undergoing financial liberalisation and policy reform, the efficiency of the use of digital finance and the deepening of the balance between quality and quantity in financial development are particularly important for economic growth. This paper investigates the utility of digital finance and financial development on total factor productivity in China using interprovincial panel data decomposing financial development into financial scale and financial efficiency; an interprovincial panel data model is used to explore the utility of digital finance on total factor productivity. This involves the collection and preprocessing of financial data, including feature engineering, and the development of an optimised predictive model. We preprocess the original dataset to remove anomalous information and improve data quality. This work uses feature engineering to select relevant features for fitting and training the model. In this process, the random forest algorithm is used to effectively avoid overfitting problems and to facilitate the dimensionality reduction of the relevant features. In determining the model to be used, the random forest regression model was chosen for training. The empirical results show that digital finance has contributed to productivity growth but is not efficiently utilised; China should give high priority to improving financial efficiency while promoting financial expansion; rapid expansion of finance without a focus on financial efficiency will not be conducive to productivity growth.

## 1. Introduction

The role of financial development in promoting economic growth has been unanimously recognised by scholars at home and abroad [1–3] and it was found that the scale and function of finance can effectively stimulate long-term economic growth as well as total factor productivity growth through their studies. The main emphasis is on a kind of guiding effect of financial development on supply, that is, with the growth rate of economic development as well as the complexity of economic structure, social demand for financial aspects will further stimulate the development of the economy, and financial development and economic growth are causally related to each other [4–6].

A vector error correction model is used to separately verify the existence of a significant positive relationship between financial development and total factor productivity. There is a large body of research literature, both domestic and international, on the utility of digital finance for economic growth [7]. An endogenous growth model based on digital finance argues that digital finance, as the main carrier of knowledge products, is an alternative to knowledge and innovation. The existence of digital finance overcomes the constraint of diminishing marginal returns to factors and makes long-term economic growth possible [8, 9]. The study points out that the long-term growth rate of the economy is directly proportional to the long-term growth rate of basic knowledge, that the ultimate variable determining the long-term growth rate of basic scientific knowledge is the stock of digital finance in the economy, and that digital finance is the real source of economic growth. Paper [10] concluded that higher education in the eastern, central, and western regions all contributes significantly to the GDP growth rate, but the contribution is distributed in a gradient from higher to lower.

The measurement of total factor productivity growth can be broadly grouped into two categories: the growth accounting approach and the econometric approach [11]. The econometric approach uses various econometric models to estimate total factor productivity, taking into account the effects of various factors in a more comprehensive manner, but the estimation process is more complex [12]. One type of econometric method is the potential output method, also known as the frontier production function method, which has been widely used in current research. These methods use changes in inputs and outputs and the displacement of the frontier production function to measure total factor productivity growth, the key to which lies in the estimation of the frontier production function and the measurement of the distance from observations to the production frontier [13]. Depending on the method of estimating the frontier production function and the distance function, the frontier production function method can be divided into two categories: First, the stochastic frontier analysis (SFA) method, of which the more popular methods are Hildreth and Houck's random coefficient panel models [14] (this is more problematic for empirical studies with small sample sizes); secondly, nonparametric data envelopment analysis (DEA).

## 2. Data Acquisition and Processing

There is a lot of noise and missing values in all types of real data, which are detrimental from the point of view of training algorithmic models. It is important to carry out the necessary preprocessing before using the data information to improve its quality and make the training of the model smoother, which is important for data mining purposes [15].

### 2.1. Feature Engineering

For machine learning, feature engineering is required to improve the performance of a model. The original dataset is the input and the relevant dataset used in the future model training process is the output, which can be used to select more desirable training features and thus achieve good results in simple structural models. The current work will address the general process of feature construction and processing, feature selection, and analysis.

Steps are as follows:

(1) First find the minimum (min) and maximum (max) of the original sample data *X*.
(2) Calculate the coefficients *k* by expressing them as follows:
  (1) $$\begin{array}{c} k=\frac{100}{\left(\max-\min\right)}. \end{array}$$
(3) The data normalized to the interval [0, 100] is obtained *y*^*∗*^ as follows:
  (2) $$\begin{array}{c} y^{*}=k\left(X-\min\right). \end{array}$$

In this paper, the data on the number of public cars per 10,000 people (×18), urban disposable income per capita (×19), and rural disposable income per capita (×20) are normalized so that these data become continuous variables in the range of [0, 100].

### 2.2. Feature Selection

Once the analysis, construction, and processing of the relevant features have been completed, feature selection is performed. Those features that have a high correlation with the target variables are selected and those that are not are eliminated [16]. The selected feature subsets are identified as the input to the model training process, resulting in a significant increase in model accuracy and performance and a corresponding decrease in training time costs.

Fitting a series of features together gives a better fit than fitting individual features, resulting in a significant increase in the predictive power of the model. However, this does not mean that more features will give better results. Random forest is an integrated learning algorithm consisting of multiple decision trees, which is easy to implement, is computationally compact, and has high performance in classification and regression and is one of the representative techniques in current integrated learning technology [17]. If the relevant features are selected by the random forest algorithm, the problem of overfitting caused by a large number of features can be effectively solved on the one hand, and the relatively minor features can be filtered out to make the prediction results more accurate on the other hand.

The key function of the random forest algorithm is to accurately calculate the importance of each feature variable. The basic principle of importance measurement is to calculate the specific contribution of each feature in each tree, to obtain its mean value, and to compare the contribution of different features [18]. The error rate of out-of-bag data is often used as an important metric for evaluation. The importance of each feature is used as an aid in the feature selection process, so that the robustness of the model is increased and the dimensionality of the features is reduced. The actual out-of-bag error rate (i.e., OOB) of each feature allows us to calculate the specific importance of the feature. The specific algorithm is described in equation:

(3) $$\begin{array}{c} {\text{FIM}}_{j}=\frac{\sum \left(\text{errOOB}2-\text{errOOB}1\right)}{N}. \end{array}$$

 Here, err OOB2 is the out-of-bag correlation error size when noise is added to feature *j* in a random way; errOOB1 is the out-of-bag correlation error size under normal conditions; *N* is the total number of trees in the random forest; *j* is feature *j*; and FIM is the actual rating of the importance of the feature. If noise is added to feature *j*, it significantly reduces the out-of-bag accuracy level, which means that the final outcome of the prediction is significantly influenced by feature *j*, and the importance of the feature is high.

## 3. Estimation of Total Factor Productivity Growth

### 3.1. Estimation Methodology

This paper draws on the nonparametric DEA-Malmquist index method of [19] to estimate total factor productivity growth in China's provinces. Assume that there are *H* agents, where the input of the *h*th agent in period *t* is *x*_*h*_′=(*K*_*ht*_, *L*_*ht*_)′, *K*_*ht*_ is the capital stock input, and *L*_*ht*_ is the labour input. Then the Malmquist index of total factor productivity growth in period *t* + 1 for the *h*th subject is

(4) $$\begin{array}{c} M_{h}^{t+1}\left(x_{h}^{\prime },y_{h}^{\prime },x_{h}^{t+1},y_{h}^{t+1}\right)={\left[\frac{D_{h}^{\prime }\left(x_{h}^{t+1},y_{h}^{t+1}\right)}{D_{h}^{\prime }\left(x_{h}^{\prime },y_{h}^{\prime }\right)}\frac{D_{h}^{t+1}\left(x_{h}^{t+1},y_{h}^{t+1}\right)}{D_{h}^{t+1}\left(x_{h}^{t},y_{h}^{t}\right)}\right]}^{1/2},\;h=1,\ldots ,H. \end{array}$$

When the total factor productivity growth index is greater than one, it means that total factor productivity growth is positive, while the opposite means that total factor productivity growth is negative.

The Malmquist index has two advantages over traditional growth accounting methods: it eliminates the need for factor price information and economic equilibrium assumptions; and it provides more comprehensive information on total factor productivity growth by decomposing it into two components: efficiency change and rate of technological progress. This method is only applicable to panel data.

## 4. Construction of a Random Forest Regression Model

The following procedure is involved in the construction of this type of model.

1. Samples are randomly drawn from the initial data set in a put-back and unweighted manner, so that each decision tree will be generated from its training set.
2. Decision tree can be constructed from each training set; no pruning is required at this point.
3. A series of decision trees together form a random forest. The prediction mean of each decision tree forms the final prediction result.

Figure 1 details the modelling process.

### 4.1. Data Sampling

For each decision tree, it corresponds to a particular training set, so the original dataset is used as the basis for forming the relevant subset of data (so that both have an equal number of decision trees) and thus the random forest is constructed. The corresponding dataset is obtained through a random sampling technique. This technique covers two different types of sampling methods: reverse and one-way.

A specific set of samples is taken from a dataset and not put back when the samples are collected; this is called nonreturn sampling. These include the random number method and the lottery method. The former is the sampling of a data set by means of a random number formation or table. In the case of nonreturn sampling, the initial dataset will continue to get smaller during the sampling process, so that there will be no duplication of samples in the subdataset. In the latter case, the entire data is numbered, the data set is homogenised, and the relevant subsets are extracted by a random method (with a capacity of *n*). Although the latter method is relatively straightforward, the difficulty of homogenisation increases when there is a large dataset, making the resulting sample unrepresentative.

### 4.2. Constructing Decision Trees

When constructing a decision tree, it is crucial to choose the random feature variables appropriately. The basic attributes associated with node splitting are called random feature variables. They are selected in order to reduce the correlation between decision trees and to improve the performance of the random forest algorithm. The random feature variables can be generated by combining input variables or by random selection. The selection process involves a number of indicators, including the Gini index, information gain ratio, and information gain. The CART algorithm is based on the Gini impurity index, which is used as the basis for determining the classification scale for effective selection.

The above process results in a number of decision trees that together form a random forest. The final result of the model is the mean of the predicted values of all the decision trees.

## 5. Empirical Analysis

### 5.1. Model Setting

Based on the claim that the level of digital finance can facilitate access to technology, the following equation for total factor productivity growth is proposed:

(5) $$\begin{array}{c} \Delta a_{it}=c+gh_{it}+m\left[\frac{h_{it}\left(y_{\max t}-y_{it}\right)}{y_{it}}\right]+\theta i, \end{array}$$

where *y*_max*t*_ represents output per capita in the technologically advanced region and *y*_*it*_ is output per capita in period *t* in region *i*. *h*_*it*_ represents digital finance in period *t* in region *i*, *a*_*it*_ represents total factor productivity, and *i* represents individual provincial fixed effects, which are included to control for possible variability between provinces [19, 20]. In this model, total factor productivity growth depends not only on the level of digital finance in the current period, but also on the interaction term between digital finance and the difference in technology levels in technology-led regions. Based on this model, the following model is developed to analyse the utility of digital finance and financial development on total factor productivity growth:

(6) $$\begin{array}{c} a_{it}=c+gh_{it}+m\left[\frac{h_{it}\left(y_{\max t}-y_{it}\right)}{y_{it}}\right]+\alpha {\text{fin}}_{it}+\beta_{j}{\text{ctrl}}_{jit}+\theta i+\varepsilon_{it}. \end{array}$$

Among them, fin_*it*_ is the level of financial development. According to the research of [21–23], the effect of financial scale and financial efficiency on the economy is different. The effect of financial scale and financial efficiency on the economy through the growth of total factor productivity should also be different. Therefore, this paper divides the level of financial development into financial scale and financial efficiency, to explore its role in the growth of total factor productivity. *c* is the control variable, which is the government intervention, the degree of economic activity, and the degree of opening to the outside world. *ε*_*ij*_ is the random disturbance term. Empirical analysis is carried out according to model (4).

Endogenous growth theory holds that digital finance is an important reason to explain total factor productivity. It has a significant impact on total factor productivity through influencing technological innovation ability, technology spillover absorption ability, and other channels.

It can be seen from Table 1 that the statistics of Kao test are statistically significant at the 1% level; that is, the original assumption that there is no cointegration relationship cannot be accepted at the 1% level. Therefore, it is considered that there is cointegration relationship between the two variable systems and regression analysis can be carried out [24, 25].

### 5.2. Empirical Results

In this paper, fixed and random effects panel data models are used.  Table 2 presents the model estimation results, where columns (1) and (2) present the utility analysis of digital finance and financial size on total factor productivity growth, and columns (3) and (4) present the utility analysis of digital finance and financial efficiency on total factor productivity growth. Hausman test *p* values are 0.9641 and 0.8420, respectively, which are both greater than 0.10; therefore, at the 10% level the original hypothesis that individual effects are correlated with explanatory variables cannot be rejected at the 10% level, so it is decided that a random effects model should be chosen instead of a fixed effects model [26, 27].

From there, the analysis is based on the model estimation results in columns (2) and (4).

The analysis focuses on the core variables to be explored in this paper, digital finance lnhit, the interaction term between digital finance and technology level differences lnhmaxit, and the impact of financial development indicators lnfscit and lnfefit on total factor productivity growth.

Column (2) presents the estimated results of the regression of digital finance and financial scale on total factor productivity growth. From the estimated results, the estimated coefficient of digital finance on total factor productivity growth is 0.0427, which is statistically significant at the 5% level; i.e., when the level of digital finance increases by 1, it will contribute to an increase in total factor productivity growth by 0.0427. Therefore, strengthening education efforts and increasing the level of digital finance are conducive to promoting an increase in total factor productivity growth, which in turn will contribute to economic growth. The interaction term between digital finance and technology level difference is negative (−0.0000984) and statistically significant at the 5% level; i.e., technology level difference shows a negative effect in the effect of digital finance on total factor productivity growth; the greater the technology level difference, the more negative the effect of the utility of digital finance on total factor productivity growth, but this negative effect is relatively small; it can be seen that the use of digital finance in China is relatively inefficient and the ability to learn new technologies is weak. The estimated coefficient of the effect of financial size on TFP growth is −0.177, which is statistically significant at the 1% level, suggesting that every 1 increase in financial size will contribute to a 0.177 decrease in TFP, possibly because state-owned enterprises receive most of the incremental financial resources due to implicit government guarantees, but do not use them effectively or even have idle funds, while the private economy, which operates more efficiently, faces a chronic shortage of capital, and the expansion of credit is also inflationary, leading to a recession [28, 29].

Column (4) presents the estimated results of the regression between digital finance and financial efficiency on total factor productivity growth. The estimated coefficient is 0.0564, which is statistically significant at the 1% level. The elasticity of financial efficiency to total factor productivity growth is 0.289, which is statistically significant at the 1% level, indicating that an increase in financial efficiency can contribute to an increase in total factor productivity growth, and an increase of 1 in financial efficiency will increase total factor productivity growth by 0.289. In addition, the contribution of financial efficiency in China (0.289) is greater than the inhibiting effect of financial size (0.177), so China should continue to carry out institutional reforms to promote financial efficiency in order to promote economic growth.

For the control variables, the results in columns (2) and (4) are generally consistent. The estimated coefficient of government expenditure on total factor productivity growth is positive, which shows that increased government expenditure is conducive to economic growth and that appropriate government intervention is conducive to healthy economic development. The estimated coefficient for investment is negative and statistically significant at the 1% level, indicating that continued higher investment is not conducive to increased efficiency in the Chinese economy, thus showing a declining trend in the marginal return to capital. The two variables of foreign development–total exports and imports and FDI–both have negative regression results in column (2), while the estimated coefficients of total exports and imports are positive and FDI remains negative in column (4), and neither is statistically significant, which is somewhat inconsistent with the fact that, according to [14], exports and imports may inhibit firms through the following channels. Firstly, domestic exporters face a latecomer disadvantage in R&D innovation in international markets, with internationally available technologies creating strong patent barriers and barriers to domestic firms' innovation, which cannot be applied unless domestic firms have a practical innovation. Secondly, international dominant enterprises suppress and control the R&D behaviour of China's export enterprises, resulting in serious “capture effect” and “lock-in effect,” which will eventually lead to a “ceiling effect” on the technological progress of export enterprises.” Therefore, the impact of international trade on total factor productivity depends on the outcome of the game between positive and negative forces, and only when the technology spillover effect is greater than the “barrier effect” can it significantly contribute to total factor productivity growth. For FDI, some scholars point out that, in places where resources are more scarce, FDI firms as dominant firms may seize the production and market resources of domestic firms, thus causing the decline of domestic firms. Therefore, FDI may have a dampening effect on total factor productivity.

### 5.3. Comparison of Model Results

The current work has used RF, SVR, and MLR methods in comparative studies. In this work, the bias of the random sampling process is effectively reduced by means of a tenfold cross-validation method, which requires the calculation of the mean value to obtain the relevant indicators for the prediction assessment. In general, the metrics used are RMSE, MSE, and MAPE. The results are given in Table 3.

In the regression models presented in the previous section, the parameters are the default parameters in the computational library and are compared with each other for the same conditions. A detailed analysis of the prediction results shows that these algorithms have generally consistent prediction results, in the following order: MLRRFSVR. The middle of the range of errors was obtained by the random forest method with an error of 22.58%, and the larger error value was obtained by the multiple linear regression method (about 38.98%). Compared to linear regression, prediction by nonlinear regression has relatively better results. It can be found that if a multiple regression correlation model is used, it will have a high training efficiency and convenience, but relatively poor nonlinear learning ability. The random forest approach (based on regression trees) has better prediction results, and the support vector machine regression approach would have better prediction results. In the current work, with a relatively small dataset and a small number of features, the advantages of the random forest approach are difficult to realize, and the factors that affect carbon productivity in practice are complex, including consumption structure, energy efficiency levels, and differences between cities (regions). By increasing the number of features, the advantages of random forests are highlighted and the accuracy of the prediction results is increased.

The current work uses the best values of the parameters as its input and then compares them with the default parameters, as shown in the data in Table 4.

Here, RF_opt and RF_def are the random forest regression model with optimal and default parameters, respectively. A detailed comparison of the above evaluation metrics shows that, for the case of optimal parameters, the errors of MAPE and RMSE are reduced by about 17.23% and 7.72%, respectively, which means that the prediction results are better than those with default values. The current work is based on the commonly used parameters of interest, and the best values are obtained by a grid search algorithm and optimised, which greatly increases the accuracy.

## 6. Conclusions

The study points out that the long-term growth rate of the economy is directly proportional to the long-term growth rate of basic knowledge, that the ultimate variable determining the long-term growth rate of basic scientific knowledge is the stock of digital finance in the economy, and that digital finance is the real source of economic growth. The role of financial development in promoting economic growth has been unanimously recognised by scholars at home and abroad. This paper examines the utility of digital finance and financial development on total factor productivity in China using interprovincial panel data. The results show that digital finance has contributed to the improvement of total factor productivity, but there is still a problem of inefficient use of digital finance in China; to this end, this paper proposes a random forest regression model with a related optimisation process. First, a training set is generated using random sampling, and a number of decision trees are constructed using a series of operations to obtain a random forest. The final result of the model is the mean of the predicted values of all the decision trees. The model is then used as the basis for regression. In the current work, the main parameters of the regression function are adjusted in order to optimise the prediction model and improve its accuracy. China should give high priority to improving financial efficiency while promoting financial expansion, which is detrimental to the growth of total factor productivity, the source of economic growth.

## Figures and Tables

**Figure 1:** Random forest regression model construction process.

**Table 1:** Panel cointegration tests for variables.

	Variable system	Kao test
dfsc	Dtfp dh dhmax dexp dinv dxm dfdi	−5.0319
dfef	Dtfp dh dhmax dexp dinv dxm dfdi	−4.7336

**Table 2:** Panel data model estimation results.

	1	2	3	4
dtfp	dtfp	dtfp	dtfp	
dh	0.0417	0.0451	0.0524	0.0587
	1.92	2.16	2.47	2.87
dhmax	−0.000906	−0.000947	−0.0000847	−0.0000874
	−2.02	−2.33	−0.84	−2.13
dfsc	−0.174	−0.1771		
	−4.43	−5.29		
dfef	0.273			0.288
	3.93	4.65		
dexp	0.215	0.223	0.218	0.221
	1.07		1.06	1.09
dinv	−4.83	−0.436	−0.528	−0.458
	−3.5	−3.56	−3.72	−3.67
dxm	−0.0145	0.00047	0.07475	0.0754
	−0.17	−0.13	0.91	0.95
dfdi	−0.0063	−0.00478	−0.00627	−0.00517
	−0.90	−0.74	−0.90	−0.76
_cons	0.00607	0.00419	0.00653	−0.00208
	0.76	0.56	0.07	−0.25
*N*	318	218	320	320
Adj. *R*^2^	0.165		0.152	
rmse	0.104	0.0098	0.105	0.009
Sman test (*p* value)	1.93	0.09647	3.43	0.8432

**Table 3:** Information on the evaluation indicators of the three models.

Regression model index	RMSE	MSE	MAPE
MLR	0.4714	0.2547	0.3874
SVR	0.7985	0.5674	0.1747
RF	1.534	2.4711	0.2257

**Table 4:** Table of results of the random forest correction model.

Model index	RMSE	MSE	MAPE
RF_opt	1.574	2.547	0.2241
RF_def	1.4527	2.1047	0.1574

## Data Availability

The experimental data used to support the findings of this study are available from the corresponding author upon request.
